The article "Hydroxyphenyl Butanone Induces Cell Cycle Arrest through Inhibition of GSK3β in Colorectal Cancer" was retracted in 2024. Reasons: signs of a paper mill; suspected computer-generated content; unreliable results or conclusions; concerns about the data.

# Hydroxyphenyl Butanone Induces Cell Cycle Arrest through Inhibition of GSK3*β* in Colorectal Cancer

**DOI:** 10.1155/2021/9981815

**Published:** 2021-07-03

**Authors:** Songyan Zhang, Yunfeng Wang, Haopeng Zhang, Chengming Sun, Shuwei Dang, Ming Liu

**Affiliations:** ^1^Department of General Surgery, The Second Affiliated Hospital of Harbin Medical University, Harbin 150086, China; ^2^Department of General Surgery, The Fourth Affiliated Hospital of Harbin Medical University, Harbin 150001, China

## Abstract

**Background:**

Colorectal cancer (CRC) is among the top three gastrointestinal malignancy in morbidity and mortality. The abnormal activation of Wnt/*β*-catenin pathway is considered to be a key factor in the occurrence and development of CRC. Novel inhibitor discovery against key factor in WNT pathway is important for CRC treatment and prevention.

**Methods:**

Cell proliferation was detected after hydroxyphenyl butanone treatment in human colorectal cancer HCT116, LOVO, and normal colonic epithelial NCM460 cells. Colony formation, cell invasion ability, and cell cycle were detected with and without GSK-3*β* knockdown.

**Results:**

Hydroxyphenyl butanone induces cycle arresting on G1-S phase of colorectal cancer cell line through GSK3*β* in Wnt/*β*-catenin pathway and inhibits malignant biological manifestations of cell proliferation, colony formation, and invasion. The inhibition in the high concentration group is stronger than that in the low concentration group, and the antitumor effect is different for different tumor cells. Under the same concentration of natural hydroxyphenyl butanone, the inhibition on normal colonic epithelial cells is significantly lower than that on tumor cells. The natural hydroxyphenyl butanone with medium and low concentration could promote the proliferation of normal colonic epithelial cells.

**Conclusion:**

This study illustrated natural hydroxyphenyl butanone as new inhibitor of GSK3*β* and revealed the mechanisms underlying the inhibitory effects in colorectal cancer.

## 1. Introduction

Colorectal cancer (CRC) is one of the most common gastrointestinal malignancy. The morbidity and mortality of CRC are among the top three malignant tumors [1–3]. Although great improvement has been achieved in diagnosis and treatment of CRC, the 5-year survival rate of CRC is still too low, and about 47.2% CRC patients showed recurrence of tumor. Recent studies have suggested that the development of CRC has a close relationship with many pathways, such as Wnt/*β*-catenin, EGFR, p53, MAPK, Notch, and RhoA/ROCK, among which Wnt/*β*-catenin pathway might be most important. The abnormal activation of Wnt/*β*-catenin pathway is considered to be a key factor in the occurrence and development of CRC [4]. In addition, Tan et al. proved that the proliferation and apoptosis of CRC cells can be inhibited by the inactivation of Wnt/*β*-catenin pathway [5].

Wnts are a series of glycoproteins related to stimulation of receptor-mediated signal transduction pathways. The enrichment of nuclear *β*-catenin is one of the most critical factors to activate Wnt pathway. After targeted for phosphorylation of the N-terminal by glycogen synthase kinase 3*β* (GSK-3*β*) at Ser33/Ser37/Tr41 residues, the cytoplasmic level of *β*-catenin is regulated by ubiquitin-mediated proteolysis. The phosphorylation of *β*-catenin by GSK-3*β* occurs in an Axin-APC complex [6, 7], during which GSK-3*β* activity presents a negative correlation with the presence of Wnt pathway [8]. *APC* is the key regulator of Wnt pathway, and mutations of *APC* are observed in at least 70% of CRCs, especially in early colonic neoplasia [9, 10]. In addition, Ashok et al. found that luteolin inhibited HCT-15 cell proliferation by downregulation of the inactive form of GSK-3*β* [11]. However, though there are many studies on Wnt/*β*-catenin pathway, its exact role in CRCs still needs more investigation.

With the increasing of old population [12, 13], the demand for low-toxic and high-efficient antitumor treatment methods is increasing. According to statistics data [14], from 1940 to 2014, more than 75% of anticancer drugs directly came from natural products. Therefore, it is of great significance to search for new effective anticancer drugs from natural products to improve the prognosis of CRC patients. Recent research also revealed that many kinds of extracts from plants (in different parts, such as barks, leaves, and fruits) have the ability of anticolon cancer cells *in vivo* or *in vitro* [15–17]. Zhang et al. showed that azoxymethane-induced upregulation of WNT/*β*-catenin pathway was prevented by genistein, which reduced colon preneoplasia in rats [18]. Reabroi et al. showed that the anticancer activity of 19-O-triphenylmethyl andrographolide involves the inhibition of Wnt/*β*-catenin signaling via a GSK-3*β*-independent pathway [19]. Aisha et al. found that xanthone extracts caused significant growth inhibition of HCT 116 colorectal carcinoma cells by upregulating the MAPK/ERK, c-Myc/Max, and p53 pathways [20].

Red raspberry (*Rubus idaeus L*.) is a kind of economical berry crop that contains numerous potential healthy compounds, such as polyphenols, flavonoids, kaurane-type diterpenoids glycosides, oleanane, sodium-type triterpenoids, glycosides, and esters [21]. Related studies have shown that red raspberry phytochemical extracts [22] had many pharmacological effects. Raspberry ketone had the ability of increase norepinephrine-induced lipolysis in white adipocytes, which could prevent and improve obesity and fatty liver [23]. The extract of red raspberry fruit showed anti-inflammatory properties to reduce the degree of bone resorption, soft tissue swelling, and osteophyte formation, preventing articular destruction in treated animals [24]. Wang et al. tested the protective effect of raspberry ketone against nonalcoholic steatohepatitis and confirmed its function in protecting kidney function, weight loss, and antialcoholic steatohepatitis [25]. Meanwhile, research on the biological activity of red raspberry leaf polyphenols showed certain effects on inhibiting human laryngeal carcinoma (HEp2) and colon adenocarcinoma (SW 480) cell lines [26]. The phytochemical extracts of red raspberry had been proved to have certain preventive effect on many kinds of malignant tumors, such as esophageal cancer [27], breast cancer [28], cervix cancer [29], and prostate cancer [30]. Experiments showed that the increasing doses of red raspberry extract could lead to inhibition of hepatocellular carcinoma [31]. Black raspberry extract had the ability of reducing acute UVB-induced inflammation which could help to prevent human skin cancers [32]. David et al. reported the anti-inflammatory effect of raspberry on DSS-induced colonic injury, which is considered to be one of the precancerous lesions of CRC [33]. Results showed a significantly increase preventive effect of CRC and ulcerative colitis. Therefore, it is speculated that the phytochemical extract of red raspberry may have broad application prospects in CRC prevention and treatment.

Red raspberry phytochemical extract is the active component of red raspberry fruit extraction. In our previous studies, we identified the extraction method and found that hydroxyphenyl butanone is the main component of red raspberry phytochemical extract, which can play a variety of antitumor effects. In this study, we aimed at revealing natural inhibitor in colorectal cancer and discovering the biochemical mechanisms of natural hydroxyphenyl butanone.

## 2. Methods

### 2.1. Preparation of Natural Hydroxyphenyl Butanone

The 4-p-hydroxyphenyl-2-butanone (pure raspberry ketone) was purified by the School of Chemical Engineering, Harbin University of Technology. For natural hydroxyphenyl butanone, fresh red raspberry was purchased from Shangzhi City, Heilongjiang Province. In the preliminary study of our research group, 100 g red raspberry/300 ml absolute ethanol (1 : 3, *w*/*V*) was mixed, homogenized by polyteron homogenizer, vacuum filtered, and evaporated at 45°C to extract the chemical extract of red raspberry. The main component was determined as raspberry ketone (4-p-hydroxyphenyl-2-butanone) by HPLC, ellagic acid, and polysaccharide. This method takes into account the effectiveness of chemical extracts of red raspberry plants and the safety of long-term human application after extraction and has been applied to the scientific research on the antihuman hepatocarcinoma effect of chemical extracts of red raspberry plants and published research papers [34, 35].

### 2.2. Cell Culture

Human colorectal cancer HCT116, LOVO, and normal colonic epithelial NCM460 cell line (from the School of Life Science and Technology, Harbin Institute of Technology) was used firstly. Then, cell culture was performed by using 1640 medium (Gibco) supplemented with 10% serum (Gibco, Grand Island, NY, USA) at 37°C-5% CO_2_ incubator.

### 2.3. CCK8 Method for Measuring Cell Proliferation

One thousand and fifty hundred cells/well in 96-well plates were plated into cells. After adhering to 200 *μ*l 1640 medium, the medium was aspirated at 0 h, 24 h, 48 h, 72 h, and 96 h, and 100 *μ*l of medium containing 10% CCK8 was added to each well. The OD value was read at a wavelength of 450 nm by a microplate reader for 4 hours. The 0 h OD value was used as the baseline, and the ratio of OD value to 0 h OD value at each time point was the cell proliferation multiplication. The cell proliferation multiple of the control group was base 1 at each time point, and the inhibition rate of each group was equal to one minus the proliferation ratio of each group/the proliferation ratio of the control group.

### 2.4. Colony Formation and Cell Invasion Ability Test

The cells were seeded at 400 cells/well in a 6-well plate and routinely cultured until each single cell clone was more than 50 cells, and crystal violet was fixed. The number of single cell clones was counted. Transwell plate (3428, costar) was evenly spread in the upper chamber, and 3 × 10^5^ cells/well were plated into the cells, and 1.5 ml of 1640 medium containing 0.5% serum was added, and 2.6 ml of 1640 medium containing 10% serum was added to the lower chamber. The cells were photographed under a crystal violet staining microscope after incubation at 37°C-5% for 24 hours. Four field of view counts were randomly selected in each group.

### 2.5. Cell Cycle Detection and Immunofluorescence

The cells cultured in adherent cells were trypsinized without EDTA, and then, the cells were collected by centrifugation, fixed in 75% ethanol at 4°C for 24 hours. PI stained for 30 min, and the cell cycle was measured by flow cytometry. After adhering to the cells on the glass plate, 4% formaldehyde was fixed, 10% triton-X100 was permeated, 5% BSA was blocked for one hour, and 0.5% BSA diluted primary antibody (#8480S, cell signaling, 1 : 100 dilution) was incubated at 37°C for 2 hours; the secondary antibody diluted with 0.5% PBS was incubated at 37°C for 30 minutes, and the nuclei were counterstained with 0.1% diluted DAPI for 5 minutes. The antifluorescence quencher was mounted and photographed under a fluorescence microscope.

### 2.6. Key Factor Protein Level Detection

The cells were counted who has the same number, and total protein was extracted by adding RIPA lysate at a concentration of 1 × 10^6^ cells/100 *μ*l, electrophoresed on SDS-acrylamide gel, and blotted onto a 0.2 *μ*m PVDF membrane. After 1 hour when 5% skim milk was sealed, 0.1% PBST was washed and then immersed in 0.1% PBST diluted primary antibody overnight; 0.1% PBST was washed, immersed in secondary antibody for 1 hour; 0.1% PBST was washed, and developer was added dropwise. Then, the ECL Western Blot Analysis System (Amersham Biosciences, Chalfont St. Giles, Buckinghamshire, UK) was involved to perform the parallel grayscale analysis.

### 2.7. Construction of Transfected Cell Lines with Downregulated Gene Expression

siRNA (Suzhou Gemma Gene) sequence is as follows:

Control group (NC)

Justice chain (5′-3′): UUCUCCGAACGUGUCACGUTT

Antisense strand (5′-3′): ACGUGACACGUUCGGAGAATT

GSK-3*β* downregulation gene group (GSK3*β*-SI)

Justice chain (5′-3′): GGACUAUGUUCCGGAAACATT

Antisense strand (5′-3′): UGUUUCCGGAACAUAGUCCTT

Human colorectal cancer HCT116 and LOVO cells were evenly plated into 6-well plates and cultured for 24 hours. The cell density was about 50%. Premixed transfection solution (containing 75 pmol of siRNA, 7.5 *μ*l of lipofectamin 2000, and 200 *μ*l of Opti-MEM medium) was added to each well. Further experiments were carried out after incubation at 37°C-5% CO_2_ for 48 hours.

### 2.8. RT-PCR

The adherent cultured cell samples were extracted with 1 *μ*g of total RNA by using TRIzol, reversely transcribed into cDNA by reverse transcription kit and subjected to RT-PCR detection using a ViiATM7 real-time PCR instrument (Applied Biosystems).

*GSK-3β* gene primer sequence is as follows:

Upstream 5′-3′: AGACGCTCCCTGTGATTTATGT

Downstream 5′-3′: CCGATGGCAGATTCCAAAGG

*GAPDH* primer sequence is as follows:

Upstream 5′-AGGCTGTGGGCAAGGTCATC-3^″^

Downstream 5′-TCAGGTCCACCACTGACACG-3′

### 2.9. Positive Control

Fluorouracil (5-fluoro-2,4(1H,3H)-pyrimidine dione, 5-FU) is a classic antitumor drug for colorectal cancer. At present, most of the chemotherapy regimens for large intestine are centered on fluorouracil or drugs that can produce fluorouracil through in vivo transformation. And it is also the commonly used positive control drug in antitumor research of colorectal cancer [3]. In this study, fluorouracil was used as the positive control of antitumor effect, and pure raspberry ketone was used as the positive control of antitumor mechanism to study the action and mechanism of red raspberry phytochemical extract on colorectal cancer cells.

## 3. Results

### 3.1. Inhibition of Natural Hydroxyphenyl Butanone on Colorectal Cancer Cell Proliferation, Colony Formation, and Cell Invasion Ability

The proliferation inhibition effects of natural hydroxyphenyl butanone, raspberry ketone, and fluorouracil were detected by CCK8 method at different times and different concentrations in colorectal cancer HCT116 and LOVO cell lines. The optimal half-inhibitory concentration of the two colorectal cancer cell lines for 72 hours culturing was determined by gradient inhibition concentration experiments and calculated by the CompuSyn software (Table 1).

The calculated half-inhibitory concentrations and 1/2 and 1/4 half-inhibited concentrations of the different red raspberry plant chemical extracts, treated for 72 hours, were calculated as the high, medium, and low experimental group concentrations according to specific colorectal cancer cell line. The half inhibitory concentration of raspberry ketone and fluorouracil, treated for 72 hours, applied as the concentration of the positive control group (Table 2).

The cell proliferation of colorectal cancer HCT116, LOVO and normal human colonic epithelial cell line NCM460 was measured at the experimental concentration. The calculated inhibition rate was as follows: 48.60 ± 6.10%/9.62 ± 5.40% for the HCT116/NCM460 high-dose raspberry group, 21.78 ± 3.79%/−2.96 ± 5.50% for the middle dose raspberry group, and 12.15 ± 3.14%/−101.30 ± 12.28% for the low-dose raspberry group, while 53.65 ± 4.60%/21.45 ± 8.57% for the raspberry ketone group and 46.48 ± 8.59%/12.06 ± 6.19% in the fluorouracil group. For LOVO/NCM460 cell lines, the results were shown as the high-dose raspberry group 54.36 ± 2.65%/−1.48 ± 5.16%, medium-dose raspberry group 15.55 ± 3.75%/−8.31 ± 8.91%, low-dose raspberry group 6.11 ± 4.00%/−52.62 ± 10.36%, raspberry ketone group 50.39 ± 2.81%/16.37 ± 6.54%, and fluorouracil group 51.64 ± 6.92%/8.69 ± 5.19%. Our analysis results showed that both of the experimental group and the positive control group have an inhibitory effect on the proliferation of colorectal cancer cell lines, and the inhibitory effect is positively correlated with the concentration of the experimental group. The experimental group and the positive control group had higher inhibitory effect on the proliferation of colorectal cancer cell lines than on normal colon cell lines. The low and medium concentration experimental group could promote the proliferation of normal colon cell lines (Figure 1(a)).

After adding experimental concentration of red raspberry phytochemical extract and raspberry ketone positive control to the medium, the number of colony formation was as follows: HCT116 control group 27 ± 3.37, high-dose raspberry group 10.5 ± 2.38, medium-dose raspberry group 20.75 ± 2.22, low-dose raspberry group 27.75 ± 3.86, raspberry ketone group 11 ± 2.16, and fluorouracil group 12 ± 2.93. For LOVO cell lines are as follows: control group 34 ± 5.42, high-dose raspberry group 8.25 ± 0.96, medium-dose raspberry group 22.25 ± 1.50, low-dose raspberry group 29.75 ± 4.03, raspberry ketone group 11.25 ± 2.99, and fluorouracil group 12.25 ± 3.86. The colony forming ability of HCT116 and LOVO cells decreased in both of the experimental group and the positive control group, and the degree of decrease was positively correlated with the concentration of the experimental group. The colony forming ability of the low concentration experimental group was close to or equal to control group (Figure1(b)). Proliferation of colorectal cancer HCT116, LOVO, and normal human colonic epithelial cell line NCM460 was measured at the experimental concentration. The calculated inhibition rate was as follows: 48.60 ± 6.10%/9.62 ± 5.40% for the HCT116/NCM460 high-dose raspberry group, 21.78 ± 3.79%/−2.96 ± 5.50% for the middle dose raspberry group, and 12.15 ± 3.14%/−101.30 ± 12.28% for the low-dose raspberry group, while 53.65 ± 4.60%/21.45 ± 8.57% for the raspberry ketone group and 46.48 ± 8.59%/12.06 ± 6.19% in the fluorouracil group. For LOVO/NCM460 cell lines, the results were shown as the high-dose raspberry group 54.36 ± 2.65%/−1.48 ± 5.16%, medium-dose raspberry group 15.55 ± 3.75%/−8.31 ± 8.91%, low-dose raspberry group 6.11 ± 4.00%/−52.62 ± 10.36%, raspberry ketone group 50.39 ± 2.81%/16.37 ± 6.54%, and fluorouracil group 51.64 ± 6.92%/8.69 ± 5.19%. Our analysis results showed that both of the experimental group and the positive control group have an inhibitory effect on the proliferation of colorectal cancer cell lines, and the inhibitory effect is positively correlated with the concentration of the experimental group. The experimental group and the positive control group had higher inhibitory effect on the proliferation of colorectal cancer cell lines than on normal colon cell lines. The low and medium concentration experimental group could promote the proliferation of normal colon cell lines (Figure 1(a)). After adding experimental concentration of red raspberry phytochemical extract and raspberry ketone positive control to the medium, the number of colony formation was as follows: HCT116 control group 27 ± 3.37, high-dose raspberry group 10.5 ± 2.38, medium-dose raspberry group 20.75 ± 2.22, low-dose raspberry group 27.75 ± 3.86, raspberry ketone group 11 ± 2.16, and fluorouracil group 12 ± 2.93. For LOVO cell lines are as follows: control group 34 ± 5.42, high-dose raspberry group 8.25 ± 0.96, medium-dose raspberry group 22.25 ± 1.50, low-dose raspberry group 29.75 ± 4.03, raspberry ketone group 11.25 ± 2.99, and fluorouracil group 12.25 ± 3.86. The colony forming ability of HCT116 and LOVO cells decreased in both of the experimental group and the positive control group, and the degree of decrease was positively correlated with the concentration of the experimental group. The colony forming ability of the low concentration experimental group was close to or equal to the control group (Figure 1(b)).

The transwell experimental cell invasion rate was detected in colon cancer HCT116 and LOVO cells with red raspberry plant chemical extracts or raspberry ketone treatment. The results of transwell were shown as HCT116 control group 27.00 ± 3.67%, high-dose raspberry group 10.50 ± 2.38%, medium-dose raspberry group 20.75 ± 2.22%, low-dose raspberry group 27.75 ± 3.86%, raspberry ketone group 11.00 ± 2.16%, and fluorouracil group 12.00 ± 2.94%; and LOVO control group 91.75 ± 14.41%, high-dose raspberry group 23.75 ± 5.12%, medium-dose raspberry group 52.00 ± 5.71%, low-dose raspberry group 76.00 ± 8.40%, raspberry ketone group 24.25 ± 3.11%, and fluorouracil group 27.25 ± 3.96%. The lower cell invasion ability was detected in the experimental group and the positive control group, and the degree of weakening was positively correlated with the concentration of the experimental group. The cell invasion ability of the low concentration experimental group was close to or equal to that of the control group (Figure 1(c)).

### 3.2. Natural Hydroxyphenyl Butanone Blocked G1-S Phase of Colorectal Cancer Cell Cycle through WNT Pathway

Applying qualitative analysis of immunofluorescence for detecting the expression of WNT pathway key proteins, *β*-catenin showed decreasing expression in the experimental group and positive control group after red raspberry phytochemical extract and raspberry ketone treatment, while *β*-catenin protein plays a regulatory role in the nucleus by binding to downstream-related nuclear factors. Furthermore, the distribution of *β*-catenin protein transferred from cytoplasm and nucleus in the control group became mainly in the cytoplasm, and the distribution in the nucleus was significantly reduced (Figure 2(a)).

Flow cytometry was applied to determine the cell cycle distribution of each group (HCT16/LOVO): G1 phase control group 41.54 ± 0.50%/38.31 ± 1.33%, high-dose raspberry group 57.78 ± 2.04%/59.22 ± 1.28%, medium-dose raspberry group 50.00 ± 0.59%/52.00 ± 2.00%, low-dose raspberry group 49.17 ± 1.34%/43.62 ± 1.63%, and raspberry ketone group 65.15 ± 0.91%/61.77 ± 1.11%; S-phase control group 51.07 ± 2.12%/50.70 ± 1.99%, high-dose raspberry 39.20 ± 1.58%/36.32 ± 1.35%, medium-dose raspberry group 46.43 ± 2.27%/43.00 ± 3.00%, low-dose raspberry group 48.66 ± 2.83%/53.85 ± 2.81%, and raspberry ketone group 23.56 ± 0.79%/30.64 ± 1.28%; and G2 control group 7.38 ± 1.70%/11.09 ± 1.58%, high-dose raspberry group 3.02 ± 0.54%/4.46 ± 1.12%, medium-dose raspberry group 2.00 ± 1.73%/5.00 ± 3.00%, low-dose raspberry group 2.17 ± 1.73%/2.53 ± 1.58%, and raspberry ketone group 11.30 ± 1.70%/7.64 ± 0.81%. The G1 phase cells in the experimental group and the positive control group increased, and the S phase cells decreased, suggesting that there is a G1-S phase cell cycle arrest; the degree of blockade is positively correlated with the concentration of the experimental group, and the concentration of the low concentration experimental group is close to or equivalent to the control group (Figures 2(b) and 2(c)).

The expressions of wnt1, wnt3a, wnt5a, *β*-catenin, CyClinD1, and CDK4 protein were downregulated in Western blot, and GSK3*β* and APC protein expressions were upregulated, resulting that WNT channel as a whole is in a state of reduced function after treatment. Red raspberry phytochemical extracts can cause the downregulation of the WNT pathway key protein *β*-catenin in the colorectal cancer cell and the decrease in the distribution of nuclei in its function region. The downregulation of the function of the WNT pathway and cell cycle-related proteins CyClinD1 and CDK4 downstream of the WNT pathway leads to cell cycle arrest (Figure 2(d)).

### 3.3. The Rescue of Inhibitory Effect of Natural Hydroxyphenyl Butanone by Blocking the WNT Pathway Key Protein GSK3*β*

The siRNA knockdown could reduce the GSK-3*β* RNA expression to 30% (HCT116 31.92 ± 7.92%, LOVO 28.52 ± 7.42%) of the control group in the colorectal cancer HCT116 and LOVO cell lines while the protein level expression is also significant downregulated (Figures 3(a) and 3(b)). After the expression of GSK-3*β* was downregulated by siRNA transfection, colorectal cancer HCT116 and LOVO cells were treated with red raspberry plant chemical extracts and raspberry ketones, WNT pathway protein constitutive proteins *β*-catenin, CyClinD1, and CDK4 on Western blot. The change from the control group is reduced (Figure 3(c)). The siRNA transfection blocking GSK-3*β* could rescue the effect of red raspberry plant chemical extracts on proteins related to cell cycle regulation downstream of GSK-3*β* in the WNT pathway. After the expression of GSK-3*β* was downregulated by siRNA transfection, the experimental concentrations of red raspberry plant chemical extract and raspberry ketone positive control were added to the medium, and *β*-catenin protein was compared with the control group by qualitative analysis of immunofluorescence. The difference in expression level could be rescued, and the difference in expression distribution in the nucleus and cytoplasm is also reduced (Figure 3(d)). Our result proved the chemical extract of red raspberry plants could affect the colorectal cancer cell cycle through the WNT pathway and exerts an inhibitory effect on the colorectal cancer cells.

As an important signaling mechanism for cell growth and development, the Wnt pathway is closely related to tumors, especially colorectal cancer. As an important transcriptional regulator in the Wnt pathway, *β*-catenin plays a significant role in the inhibition of malignant expression of tumor cells through LEF/TCF and other pathways with its increase in expression and import to nucleus. This study showed that the phytochemical extracts of raspberry and raspberry ketone could downregulate the expression of Wnt pathway protein and reduce the nuclear import of *β*-catenin. The use of siRNA to blocking the Wnt pathway was significantly weakened, indicating that the phytochemical extracts of red raspberry plants and raspberry ketone exert an antitumor effect through the Wnt pathway in colorectal cancer cell lines (Figure 4).

## 4. Discussion

Our group determined the mature method of phytochemical extracts of red raspberry plants through preliminary research and found that the phytochemical extracts of red raspberry plants can inhibit the malignant manifestations of human hepatocellular carcinoma through PTEN/AKT pathway [19]. Studies have shown that raspberry ketone can inhibit the proliferation of a variety of tumor cells including colorectal cancer and lead to cell cycle G1-S phase arresting [36]; there are reports that raspberry powder can reduce the number of large intestinal abnormal crypt foci (ACF) induced by oxidation Azomethane (AOM) [37] and reduce the intestinal tumor number of APCmin/+ mice and inhibit cell proliferation activity of it [38], but the mechanisms of these effects produced by raspberry powder or raspberry ketone are not fully understood. The effects and mechanisms of phytochemical extracts of red raspberry on colorectal cancer cells are still lacking in related research, and there are no related reports whether the antitumor mechanism of raspberry phytochemical extracts and pure raspberry ketones in the above studies is exactly the same.

This study showed that the phytochemical extracts of raspberry plants and raspberry ketone can cause cell cycle G1-S arresting of colorectal cancer HCT116 and LOVO cells through Wnt pathway, inhibiting the proliferation, colony formation, and invasion. The progression of the cell cycle is tightly regulated by a complex network of cyclins, CDKs, and transcription factors at several irreversible regulatory points. The cell cycle is regulated by the CyclinD1/CDK4 complex in the early G1 [39]. CyclinD1/CDK4 is one of the important downstream regulatory pathways of the Wnt pathway, and its downregulation of expression can lead to cell cycle G1-S phase arresting. This study demonstrates that raspberry phytochemical extracts and raspberry ketones can cause cell cycle G1-S arresting by downregulating the expression of CyclinD1/CDK4 protein in colorectal cancer cell lines.

As a promoter of the Wnt signaling pathway, the Wnt family contains 14 proteins. This study found that red raspberry plant chemical extracts and raspberry ketones can cause downregulation of Wnt1, Wnt3a, and Wnt5a proteins, suggesting that it may have an inhibitory effect on multiple proteins of the Wnt family. Because the raspberry phytochemical extract and raspberry ketone may cause the downregulation of multiple Wnt family proteins, it is not suitable to verify the effect on the Wnt pathway by blocking a single Wnt family protein alone. In this study, the next level of the signal protein GSK-3*β* of the Wnt protein in the Wnt pathway was blocked for study.

Because we did not find an antitumor drug that is widely recognized and has the same antitumor mechanism as the chemical extract of the red raspberry plant, as a positive control, we chose a low concentration classic antitumor drug fluorouracil of colorectal cancer as a positive control for the cell phenotype to express the inhibition of chemical extracts of red raspberry plants on colorectal cancer cells. The mechanism of action of fluorouracil and red raspberry phytochemical extracts on colorectal cancer tumor cells was different in the cell cycle and Wnt pathway. It should not be used as a positive control. We only used pure raspberry ketone as a positive control.

Currently, clinically widely used colorectal cancer antitumor drugs such as platinum, paclitaxel, and fluorouracil are toxic to normal cells while exerting a killing effect on tumor cells. In this experiment, when the half-inhibitory concentration of tumor cells was reached, the inhibitory effect of chemical extracts of red raspberry on normal colon cells was weaker than that of fluorouracil. Under the same experimental concentration, proliferation inhibition of colorectal cancer HCT116 and LOVO cell lines exerted by chemical extracts of raspberry plants and raspberry ketone was significantly stronger than that of normal colonic epithelial cells. The chemical extracts of red raspberry in the low-intensity experimental group promoted the proliferation of normal colonic epithelial cells, suggesting that the inhibitory effect of chemical extracts of red raspberry on colorectal cancer cells may be a selective antitumor effect, which may be less toxic or even have a certain cytoprotective effect on normal colon tissue.

In the macrolevel, as a kind of widely used of raspberry fruit and functional food, its function mainly displays in the traditional medicine in the regulation of the body function, rather than the direct toxic effect of tumor; red raspberry has certain protective effect on normal colon tissue, which may be the macroeffect of microreaction in cell experiments. In terms of the microscopic molecular mechanism, this study found that red raspberry phytochemical extracts had inhibitory effects on Wnt pathway activity of colorectal cancer cells, and abnormal Wnt pathway as an important characteristic of colorectal cancer cells has been recognized as a result. There was no obvious abnormal activation of Wnt pathway in normal colon cells, which may be part of the reason why the chemical extract of red raspberry had weak toxicity and even certain protective effect on normal colon tissues. Of course, more detailed molecular mechanisms require a lot of further research is also one of the directions of further research.

Extraction pure raspberry ketone is difficult and expensive, and there is no research on the safety of drugs in humans. The chemical extract of red raspberry plant can cause the inhibition of colorectal tumor cells similar to pure raspberry ketone, and as a widely consumed food extract, its safety in human application is fully guaranteed. This study shows that the chemical extract of red raspberry has broad application prospects as a functional food against colorectal cancer. Of course, the conversion to clinical applications requires a large number of animal and human trials.

## Figures and Tables

**Figure 1:** Effect of natural hydroxyphenyl butanone on proliferation, colony formation, and invasion of colorectal cancer HCT116 and LOVO cells. (a) Inhibition rate of chemical extracts of red raspberry with different concentrations, raspberry ketone, and fluorouracil on colorectal cancer HCT116, LOVO cells, and normal colonic epithelial NCM460 cells. (b) The effects of the chemical extracts of red raspberry with different concentrations, raspberry ketone, and fluorouracil on the colony formation of colorectal cancer HCT116 and LOVO cells. (c) Effects of different concentrations of red raspberry phytochemical extracts, raspberry ketone, and fluorouracil on colorectal cancer HCT116 and LOVO cell invasion ability. ^∗^*p* < 0.05; #*p* > 0.05.

**Figure 2:** The effect of the cell cycle of HCT116 and LOVO in colorectal cancer and *β*-catenin raised by the chemical extract of red raspberry on expression and localization in cells and Wnt pathway. (a) Effects on expression and localization of *β*-catenin in cells with different concentrations of red raspberry phytochemical extracts and raspberry ketone. (b, c) Effects of different concentrations of red raspberry phytochemical extracts and raspberry ketone on cell cycle. (d) Effects of different concentrations of red raspberry phytochemical extracts and raspberry ketone on the expression of Wnt pathway proteins. ^∗^*p* < 0.05; #*p* > 0.05.

**Figure 3:** The effect of HCT116 and LOVO cells in colorectal cancer downregulated by GSK3*β* expression and *β*-catenin raised by the chemical extract of red raspberry on expression and localization in cells and Wnt pathway. (a) GSK3*β* expression downregulated RT-PCR detection. The expression level of GSK3*β* mRNA in the HCT116 transfected group was 31.92 ± 7.92% of that in the control group and that in the LOVO transfected group was 28.52 ± 7.42% of that in the control group by RT-PCR detection. (b) Western blot detection of downregulated levels of GSK3*β* expression. GSK3*β* mRNA expression level in the HCT116 transfected group was 29% of that in the control group by Western blot analysis and was 41% in the LOVO transfected group of that in the control group. (c) Under the same experimental conditions, effects of chemical extracts of raspberry with different concentrations and raspberry ketone on the Wnt pathway of colorectal cancer HCT116 and LOVO cells with Si-RNA transfection downregulated GSK3*β* expression. (d) Under the same experimental conditions, effects of different concentrations of red raspberry phytochemical extracts and raspberry ketone on the expression and localization in cells of *β*-catenin in Si-RNA transfection colorectal cancer HCT116 and LOVO cells downregulated by GSK3*β* expression. ^∗^*p* < 0.05.

**Figure 4:** Effect of chemical extracts of raspberry plants on the Wnt pathway.

**Table 1:** Half inhibition concentration.

	Half inhibitory concentration	
	HCT116	LOVO
Red raspberry phytochemical extract	27 mg/ml	17 mg/ml
Natural hydroxyphenyl butanone	190 *μ*g/ml	174 *μ*g/ml
Fluorouracil	0.7 *μ*g/ml	0.4 *μ*g/ml

**Table 2:** Concentration of the experimental group and positive control group for 72 hours.

Groups	HCT 116	LOVO
Red raspberry extract high concentration (HRB)	27 mg/ml	17 ml/ml
Red raspberry extract medium concentration (MRB)	13.5 ml/ml	8.5 mg/ml
Red raspberry extract low concentration (LRB)	6.25 mg/ml	4.25 mg/ml
Ketone (PRB)	190 *μ*g/ml	174 *μ*g/ml
Fluorouracil (5-Fu)	0.7 *μ*g/ml	0.4 *μ*g/ml

## Data Availability

The datasets used and/or analysed during the current study are available from the corresponding author on reasonable request.
